# Molecular Mechanism of Gas Anesthetics on the Invasion, Metastasis, and Chemosensitivity of Osteosarcoma Cells

**DOI:** 10.1155/2021/6000385

**Published:** 2021-11-03

**Authors:** Qian Zhao, Jianyong Yan, Wen Li, Ye Yang, Lu You, Chenguang Qin

**Affiliations:** ^1^Department of Anesthesiology, Guizhou Provincial People's Hospital, Guizhou, China; ^2^Department of Anesthesiology, Guizhou Provincial Orthopaedic Hospital, Guizhou, China

## Abstract

**Background:**

Osteosarcoma is one of the most prominent bone cancers which has a predominant occurrence in children and adolescents. This study is focused on determining the effects of treatment of gas anesthetics on invasion, metastasis, and chemosensitivity in the progression of osteosarcoma cells. *Material and Methods*. The biological effects of the common gas anesthetics—desflurane, isoflurane, and sevoflurane—on osteosarcoma cells were studied and compared. The biological assays were performed for analysis of cell migration and proliferation.

**Results:**

Isoflurane and sevoflurane have shown significant inhibition in the osteosarcoma cells at clinically relevant concentrations. Desflurane has shown less potent action on cell migration and inhibition. All three gas anesthetics have shown inhibition in cell proliferation. The effective antiproliferative action was at a clinically significant dose. At low millimolar concentrations, cell apoptosis was moderately affected. Drug combination analysis with chemotherapeutic drugs showed relevant inhibition in cell migration. All three agents showed significant augmentation of chemotherapeutic drugs in suppression and inhibition of inducing apoptosis. The antimigration action is likely to affect the PI3K/AKT pathway and IGF-1.

**Conclusion:**

The study demonstrates the proposed mechanisms of gas anesthetics and their differential effects on osteosarcoma cells and their survival, migration, growth, and chemosensitivity.

## 1. Background

Osteosarcoma has a predominant occurrence in children and adolescents and is the primary most common bone cancer. The survival rates were recorded as more than 60% in cases of nonmetastatic osteosarcoma. The dominance of this disease is that it aggressively develops metastases which affect the long-term survival chances of osteosarcoma patients. Hence, it is difficult to understand the mechanism involved in metastasis of osteosarcoma patients. Understanding this will help in the development of future therapies. Using sevoflurane as an anesthetic in cancer surgery is common. Hence, brief information on these anesthetics on osteosarcoma cells is available [1]. Using surgical resection combined with adjuvant therapies is very effective in the treatment of osteosarcoma [2]. The survival rate in osteosarcoma has increased to 65-75% [3, 4]. The 5-year survival rate of patients is extremely low in patients showing metastasis and recurrence [5].

General anesthetics administered during the process of surgery can lower the body temperature and increase the threshold for vasoconstriction response [6]. Nowadays; gas gradually shows its therapeutic potential in many diseases, such as cardiovascular diseases and cancers [7]. Although they have been widely used, the mechanism of how they induce and maintain anesthesia has not been explained.

## 2. Methods

### 2.1. Drugs

Gas anesthetics desflurane, isoflurane, and sevoflurane were bought from Kent Scientific, USA. Paclitaxel and 5-fluorouracil were bought from Sigma, USA.

### 2.2. Cell Lines

U2OS and Saos-2 are the cells lines of human osteosarcoma which were purchased from Sigma Aldrich, USA. U2OS and Saos-2 cells were cultured in IMDM (Iscove's modified Dulbecco's medium) with 100 U/ml benzyl penicillin: 100 *μ*g/ml streptomycin solution and 10% (*v*/*v*) inactivated fetal bovine serum. The temperature for the solution was maintained at 37°C in a humidified incubator with 5% CO_2_. Insulin-like growth factor-1 was obtained from Sigma Aldrich, USA. 25 ng/ml IGF-1 was added to the media along with desflurane, isoflurane, and sevoflurane treatments, respectively, for activation of the PI3K/AKT pathway.

#### 2.2.1. Treatment with Gas

Cells were cultured at 37°C in a humidified incubator with desflurane, isoflurane, and sevoflurane.

### 2.3. Measurement of Proliferation

With 50% confluency, cells were selected for a 96-well plate for each anesthetic. Desflurane, isoflurane, and sevoflurane were added to cell plates on the next day and the chemotherapeutic drug combination. Post 72 hours of incubation, the activity of cell proliferation was determined via the BrdU Cell Proliferation Assay Kit (Sigma Aldrich, USA).

### 2.4. Measurement of Apoptosis

A 6-well plate was used for cells having 50% confluency. Various agents were added to the culture plates the next day. The agents added were various inhalational anesthetics and chemotherapeutic drug combinations. 72 hours post incubation, trypsin was added to harvest the cells for apoptosis using Annexin V Apoptosis Detection Kits (Elab Science), and Cytomics FC500 Flow Cytometer (Beckman Cell Counter, Select Science, UK) was used for analysis.

### 2.5. ELISA

Cells were incubated with respective drugs for a duration of 24 hours, harvested, and then homogenized with the help of standard protocol. Using PBS, the cell lysates were adjusted at likely concentrations. The activity of IGF-1 was analyzed with cell lysates and determined with the help of PI3K/AKT pathway Activation IGF-1 Assay Kits, respectively (Universal Biologicals, UK). At 490 nm absorbance, the active levels of IGF-1 and PI3K/AK were measured. The marker of oxidative DNA damage 8-OHdG (8-hydroxydeoxyguanosine) was measured at 450 nm absorbance. The OxiSelect™ Oxidative DNA Damage ELISA Kit (BioScience, UK) was used for the study; hence, the reagents and protocols were used as mentioned by the kit manufacturer.

### 2.6. Immunofluorescence

Cells were fixated in PBS with 4% paraformaldehyde at room temperature for fifteen minutes for U2OS and Saos-2 (Sigma Aldrich, USA). Images were taken from the Nikon E800 scope.

### 2.7. Statistical Analysis

Data analysis was performed using GraphPad Prism 6.0 software from La Jolla, USA. The data for experiments was represented as the mean ± S.D.(standard deviation). Using one-way ANOVA or unpaired Student's *t*-test, the *P* values were determined in treated groups. Bonferroni's multiple comparison test was used as a post hoc test. *P* < 0.05 was considered statistically significant.

## 3. Results

There are variable effects of inhalational anesthetics on osteosarcoma cell migration. The represented pictures are from the cell migration assay. U2OS and Saos-2 were treated with the control group and three anesthetics individually at 100 *μ*M: desflurane, isoflurane, and sevoflurane. Quantification of cell migration was done using software which showed a degree of inhibition on the osteosarcoma cells. Experiments were performed thrice for appropriate results.

## 4. Discussion

The variable effects of desflurane, isoflurane, and sevoflurane in osteosarcoma cells were studied for migration. The effects of inhalational anesthetics were analyzed by a migration assay using U2OS and Saos-2, as both U2OS and Saos-2 are cell lines for human osteosarcoma which showed significant inhibit migration in sevoflurane and isoflurane. In both isoflurane and sevoflurane, nearly 60% inhibition of migration was noted for both U2OS and Saos-2 cells whereas desflurane caused less than 20% inhibition (Figure 1). Hence, the results obtained from isoflurane and sevoflurane were more potent in inhibiting the migration of osteosarcoma cells. Additionally, U2OS and Saos-2 cells responded to desflurane in a different manner [8].

In the inference of the study, we want to say that the demonstration of findings for the inhibitory effects of inhalational anesthetics for osteosarcoma cells was noted (Figure 2). The mechanisms involved in the action are mainly due to the inhibition of the PI3K/AKT signaling pathway.

The study has shown that various surgical procedures may increase the chances of invasion and migration of cancer cells; hence, it promotes their ability to disseminate in that duration [9]. Hence, treatment with desflurane, isoflurane, and sevoflurane [10, 11] plays a crucial role in reducing the tumor recurrence postsurgery. It is crucial to choose the appropriate anesthetic for the surgical process in operating a tumor. The anesthesias have showed inhibition in the properties of migration, proliferation, and metastasis of cancer cells. New approaches can be selected on understanding the selective molecular mechanisms of anesthesia for cell proliferation and migration. This may lead to the establishment of more paths for new approaches in the treatment of osteosarcoma. The study concludes with the state that the inhalational anesthetics inhibit cell invasion, proliferation, and migration by inactivating the PI3K/AKT pathway (Figure 3). Hence, out of the three inhalational anesthetics chosen for the study, sevoflurane was the most efficient anesthesia in controlling osteosarcoma spread, hence must be clinically used as a suitable choice of drug in operation.

In order to analyze the efficacy of chemotherapy in osteosarcoma cells, we experimented the combination of studies by using gas anesthetics along with the combination of 5-FU and paclitaxel—commonly used chemotherapeutic drugs. Combination therapy of anesthetics with chemotherapeutic agents has shown around 55% inhibition in survival, proliferation, and migration (Figure 4). We found in the study that sevoflurane or isoflurane with 5-FU or paclitaxel was effective significantly in the inhibition of migration of osteosarcoma cells as compared to paclitaxel or 5-FU alone.

## 5. Conclusion

In some retrospective studies, it was found that the role of inhalational anesthetics reduced tumor metastasis and its reoccurrence. But large clinical trials and randomized trials are required on long-term outcomes in osteosarcoma studies. This will further complement in the understanding of the mechanisms involved.

## Figures and Tables

**Figure 1:** Fluorescence cell photomicrograph of exposed cells to desflurane, isoflurane, and sevoflurane. Apoptotic bodies can be seen.

**Figure 2:** Differential effects of inhalational anesthetics (desflurane, isoflurane, and sevoflurane) on osteosarcoma cell migration.

**Figure 3:** Relative comparison of BrdU in each group in comparison to the control group in cell growth and survival: (a) the relative BrdU level of cell groups; (b) the proportion of the apoptosis in each cell group. ^∗^*P* < 0.05, ^∗∗^*P* < 0.01, and ^∗∗∗^*P* < 0.001, as compared to the control group.

**Figure 4:** Relative comparison of osteosarcoma cells in migration, growth, and survival. A comparative analysis was done for control groups and all groups. The differential combination effects of inhalational anesthetics were studied on osteosarcoma cell migration, growth, and survival. The differential effects on the inhibition of growth were analyzed by (a) isoflurane and sevoflurane which significantly augmented the effects of 5-FU and paclitaxel in reducing the osteosarcoma cell migration. All the anesthetics amplify the action of 5-FU and paclitaxel by reducing osteosarcoma cells in inhibiting proliferation. (b) In induction of apoptosis, (c) desflurane, sevoflurane, and isoflurane were used in the proliferative assay. All were also used in combination forms for studying migration, proliferation, and apoptosis. ^∗^*P* < 0.05, ^∗∗^*P* < 0.01, and ^∗∗∗^*P* < 0.001, as compared to paclitaxel or 5-FU alone. Experimentation was performed three times for accurate results.

## Data Availability

The data used to support the findings of this study are available from the corresponding author upon request.
